# Progesterone and Src Family Inhibitor PP1 Synergistically Inhibit Cell Migration and Invasion of Human Basal Phenotype Breast Cancer Cells

**DOI:** 10.1155/2015/426429

**Published:** 2015-05-17

**Authors:** Mingxuan Xie, Li Zhou, Xi Chen, Lindsey O. Gainey, Jian Xiao, Mark S. Nanes, Anji Hou, Shaojin You, Qiong Chen

**Affiliations:** ^1^Department of Geriatrics, Xiangya Hospital, Central South University, 87 Xiangya Road, Changsha, Hunan 410008, China; ^2^Department of Respiratory, Xiangya Hospital, Central South University, 87 Xiangya Road, Changsha, Hunan 410008, China; ^3^Laboratory of Cancer Experimental Therapy, Atlanta Research & Educational Foundation (151F), Atlanta VA Medical Center, 1670 Clairmont Road, Decatur, GA 30033, USA; ^4^Department of Oncology, Shanghai Seventh People's Hospital, 358 Datong Road, Pudong New District, Shanghai 200137, China; ^5^Medical Service, Atlanta VA Medical Center and Division of Endocrinology, Metabolism, and Lipids, Department of Medicine, Emory University School of Medicine, Decatur, GA 30033, USA

## Abstract

Basal phenotype breast cancer is one of the most aggressive breast cancers that frequently metastasize to brain. The role of sex hormones and their receptors in development of this disease is largely unclear. We demonstrated that mPR*α* was expressed at a moderate level in a brain metastatic BPBC cell line MB231Br, which was derived from the parent mPR*α* undetectable MB231 cells. It functioned as an essential mediator for progesterone induced inhibitory effects on cell migration of MB231Br and, when coincubated with PP1, synergistically enhanced the progesterone's inhibitory effect on cell migration and invasion *in vitro*. Progesterone and PP1 cotreatment induced a cascade of molecular signaling events, such as dephosphorylation of FAK, downregulation of MMP9, VEGF, and KCNMA1 expressions. Our *in vitro* study demonstrated that mPR*α* was expressed and functioned as an essential mediator for progesterone induced inhibitory effects on cell migration and invasion in BPBC cells. This inhibitory effect was enhanced by PP1 via FAK dephosphorylation, MMP9, VEGF, and KCNMA1 downregulation mechanisms. Our study provides a new clue toward the development of novel promising agents and pathways for inhibiting nuclear hormonal receptor-negative and endocrine-resistant breast cancers.

## 1. Introduction

Current antihormonal therapies are frequently used for the treatment of hormone receptor positive breast cancers (i.e., estrogen receptor alpha and/or nuclear progesterone receptors, ER+ and/or PR+). For ER+ breast cancers, antiestrogen therapies (such as tamoxifen and anastrozole) are often effective, both in primary and in metastatic settings. The status of PR expression is used with ER to indicate potential effectiveness of antiestrogen therapies since the majority of breast cancers express ER and PR concurrently, even though PR may have independent predictive value for breast cancer [1, 2]. Previous studies with large-scale data sets found that ER+/PR− breast cancers do not respond as well as ER+/PR+ cancers to selective ER modulators [2]. It was proposed that patients with PR− breast cancer may receive a substantially better response from anastrozole rather than tamoxifen (compared to those with PR+ breast cancer) [1]. Synthetic progestin has been listed as a second line anticancer agent in “The NCCN Guidelines” (Version 1.2012 Breast Cancer, page 113). For example, megestrol acetate (MA) is used as an optional therapeutic agent for postmenopausal patients [3, 4] and medroxyprogesterone acetate (MPA) is often prescribed for treatment of metastatic breast cancer [5]. In clinical practice, cases of successful combination of MPA and chemotherapy are frequently reported in breast cancer patients with various distant metastases, including bones [6, 7], liver [8, 9], and lung [10]. For treatment of human basal phenotype breast cancer (BPBC) or triple negative breast cancer (TNBC), however, current hormonal therapies may not be appropriated since these cancers are resistant to commonly used antihormonal agents [11, 12]. Great attention has been focused on discovering new molecular targets for development of novel therapeutic tools against these cancers.

The role of progesterone (P4) on breast cancer development remains controversial. In premenopausal patients, the sex hormonal milieu in the late stage of menstrual cycle has been associated with the lowest metastatic potential, both in human breast cancer [13, 14] and in rodent mammary tumors [15, 16]. Sivaraman and Medina demonstrated that P4, when used with estrogen (E2), has a protective role against mammary tumorigenesis* in vivo* [17, 18]. The Multiethnic Cohort and Women's Health Initiative Trials, however, reported that postmenopausal women receiving estroprogestin therapy are at an increased risk of breast cancer compared with those receiving estrogen alone, supporting the concept that P4 may contribute to the development of breast cancer [19, 20]. Differing results have also been reported for the effect of P4 on breast cancer cells* in vitro*. Depending upon the experimental cell model, cell context, and duration of treatment, P4 can elicit either cancer promotion or cancer protective effects on breast cancer cells [21]. For example, P4 induced cell growth and migration of T47D cells, an ER+ and PR+ human breast cancer cell line [22], but it inhibited proliferation of MDA-MB468 (MB468) cells, a human BPBC cell line with strong membrane progesterone receptor alpha (mPR*α*) expression [23]. In another human BPBC cell line MDA-MB231 (MB231), which was negative for both PR and mPR*α* receptors, P4 induced no response in cell proliferation. Introduction of mPR*α* cDNA into these cells rescued inhibition of cell proliferation by P4 [23], indicating that the P4 → mPR*α* signaling pathway played an essential role in controlling cell proliferation of human BPBC cells [23].

Progesterone exerts rapid nongenomic actions and these nonclassical actions usually take several minutes to half an hour to act [24, 25]. Extranuclear activity has been demonstrated for nuclear PR, especially PR-B, which involves the binding of the SH3 domain of Src and rapidly activates downstream MAPK/Erk1/2 [26]. P4 also exerts actions in cells and tissues naturally devoid of PR, such as T-lymphocytes, platelets, and rat corpus luteum [27–29]. Furthermore, potent PR agonist (i.e., R5020) and PR antagonist (i.e., RU486) showed little or no effect on P4's nongenomic actions [24, 30, 31]. This evidence lends strong support to the existence of membrane-bounded progesterone receptors. Recently, cell membrane hormonal receptors, such as mPR family (*α*, *β*, *γ*) and progesterone membrane receptor component-1 (PGMRC1), were demonstrated to be functional in breast cancer [32, 33]. It was reported that rapid responses are triggered by P4 binding to membrane receptors (i.e., mPR*α*) [34–36], subsequently inducing a series of alterations in secondary messenger pathways through activation of pertussis toxin-sensitive inhibitory G-proteins, to activate MAPK/Erk 1/2 pathway [32, 33, 37, 38]. We recently reported that the signaling cascade of P4 induced mesenchymal repression is mediated through caveolae bound signaling molecules, namely, Cav-1, EGFR, and PI3K. We also observed that one of the Src family kinase inhibitors [39–41] (4-amino-5-(4-methylphenyl)-7-(t-butyl)pyrazolo[3,4-d]-pyrimidine, or PP1) blocked the P4's action on expression of occludin and E-cadherin (epithelial phenotypes) but not on the expression of snail and fibronectin (one of the mesenchymal phenotypes) [23]. The roles of Src pathway in the P4/mPR*α* induced epithelial to mesenchymal transition (EMT) relevant signaling pathways remain to be explored in human BPBC cells.

Basal phenotype breast cancer (BPBC) is one of the most malignant breast cancers accounting for 15% of all breast cancers, and recent studies show that these cancers are often associated with brain metastasis [42, 43]. Unfortunately there is no well accepted mechanism that can explain how this brain metastatic potential is being developed in human BPBC cancers, and understanding this mechanism is essential for development of novel therapeutic tools for treatment of BPBC. MB231 is classified as a basal phenotype breast cancer cell line [44]. By a series of* in vivo* selections in mice, the populations with distinct brain metastatic tropisms were isolated [45, 46]. The brain metastatic derivative MB231 cell line (MB231Br) develops brain metastasis in 100% of mice and has served as the mainstay of most brain metastasis studies [47, 48]. It was reported that MB231Br cells have increased invasiveness through both Matrigel and blood-brain barrier (BBB) but decreased proliferation rate when compared with parental MB231 cells [49]. Genome-wide expression analysis suggested alternations in the gene expression profile of 243 genes in MB231Br cells as compared with the parent line [50]. In this study, we found that the expression of mPR*α* was upregulated in MB231Br cells and thus wondered if the upregulated mPR*α* is functional and can be used as a molecular target for modulating cell biological behavior of human BPBC cancers.

## 2. Material and Methods

### 2.1. Antibodies and Pathway Inhibitors

RU486 (MIF), AG1498, wortmannin, rapamycin, and pyrazolopyrimidine compound (PP1) were purchased from EMD Chemicals (Gibbstown, NJ, USA). BpV (phen) was from Thermo Fisher Scientific (Pittsburgh, PA, USA). Anti-mPR*α* goat polyclonal IgG, anti-MMP9 goat polyclonal IgG, anti-GAPDH goat polyclonal IgG, anti-mPR*α* blocking peptide, donkey anti-goat IgG-HRP, goat anti-rabbit IgG-HRP, and anti-mouse IgG were purchased from Santa Cruz Biotechnology (CA, USA). Anti-VEGF polyclonal antibody was from Abcom (Cambridge, MA, USA). Anti-KCNMA1 rabbit polyclonal antibody was from Millipore (Billerica, MA, USA). Anti-FAK rabbit polyclonal and anti-p-FAK rabbit polyclonal IgG were from Cell Signaling (Danvers, MA, USA). P4-BSA-FITC conjugate and anti-*α*-tubulin mouse monoclonal IgM were purchased from Sigma (St. Louis, MO, USA).

### 2.2. Cell Culture

The human breast cancer cell lines MDA-MB468 (MB468) and MDA-MB231 (MB231) were obtained from the American Type Culture Collection (Rockville, MD, USA). These cell lines are negative for ER, PR, and Her-2 and are classified as “basal phenotype A” breast cancer cells [15]. The brain seeking MB231 cell line (MB231Br) was a gift from Dr. Yoneda, which was established by six successive rounds of* in vivo* selection and* ex vivo* culture from parental MB231 cells [47]. These breast cancer cells were cultured in DMEM (Mediatech, VA, USA) containing 10% FBS, 100 U/mL penicillin, and 100 *μ*g/mL streptomycin (Gibco, Carlsbad, CA, USA) in a humidified incubator at 37°C with 5% CO_2_.

### 2.3. Transfection of mPR*α* cDNA Plasmid

Transfection was performed as previously described [23]. Briefly, MB231 cells were cultured and split when the cell confluence reached approximately 90%. The human mPR*α* cDNA constructed in a pUC-based plasmid with CMV promoter (pBK-CMV) vector [30] was purified and then transfected into the cells using Lipofectamine 2000 reagent following the manufacturer's instructions (Invitrogen, Carlsbad, CA, USA).

### 2.4. RT-PCR Assay

Total RNA was extracted using TRIzol (Invitrogen, Carlsbad, CA, USA) and concentrations of RNA were determined using a NanoDrop2000 Spectrophotometer (Thermo Scientific, USA). Reverse transcription for synthesizing cDNA was carried out using the Quantitect Reverse Transcription Kit (Qiagen, Valencia, CA, USA). PCR amplification (35 cycles of 95°C for 20 sec, 58°C for 30 sec, and 72°C for 20 sec) was conducted in a total volume of 25 *μ*L using the GoTaq Hot Start Green Master Mix (Promega, Madison, WI, USA). Following PCR amplification, 25 *μ*L of the samples was separated via electrophoresis on a 1.5% agarose gel. The primers used for PCR amplification were mPR*α*-(5′-CCT GCTGTGTGATCTTAG-3′ and 5′-CGGAAATAGAAGCGCCAG-3′) [31], 18-S-(5′-GTTGGTTTTCGGAACTGAGGC-3′ and 5′-GTCGGCATCGTTTATGGTCG-3′) [51].

### 2.5. Immunoblotting Assay

Western blot assays were performed as described previously [23]. After treatment with or without P4 and/or diverse pathway inhibitors, the growth-arrested cells were lysed with 500 *μ*L ice-cold lysis buffer (50 mM HEPES, 5 mM EDTA, 50 mM sodium chloride, pH 7.4), 1% Triton X-100, protease inhibitors (10 *μ*g/mL aprotinin, 1 mM phenylmethylsulfonyl fluoride, and 10 *μ*g/mL leupeptin), and phosphatase inhibitors (50 mM sodium fluoride, 1 mM sodium orthovanadate, and 10 mM sodium pyrophosphate). Cell lysates (30 *μ*g) were separated using SDS-PAGE and transferred to nitrocellulose membranes, blocked for one hour in TBS buffer containing 5% nonfat dry milk and 0.1% Tween 20, and incubated overnight with primary antibodies at proper dilutions. After incubation with secondary antibodies, proteins of interests were detected by ECL chemiluminescence. Image J (http://rsb.info.nih.gov/ij/) was used for image analysis and quantitative data was normalized with the reference proteins (i.e., GAPDH or *α*-tubulin) or calculated as ratios of phosphor protein/total protein when the reference proteins were the same.

### 2.6. Localization of P4-BSA-FITC Binding Sites on MB231Br Cells

Breast cancer cells were cultured in chamber slides and exposed to 100 nM P4-3-(O-carboxymethyl) oxime-BSA-FITC (P4-BSA-FITC) for 30 min in serum-depleted medium [24]. Cells were then washed with PBS buffer, fixed by 10% buffered formalin, counterstained with DAPI, and observed under a confocal microscope (Olympus FV1000, Tokyo, Japan) using an oil objective lens (×60).

### 2.7. Cell Proliferation Assay

Cell proliferation assay was performed using MTT kit (Invitrogen, CA, USA) [52]. Cells were seeded in a 96-well plate in 100 *μ*L of culture medium with or without the compounds to be tested and incubated for 16 hrs at 37°C. MTT labeling reagent (1 *μ*L of stock solution) was added to the designated wells and continually incubated for 4 hrs. The supernatant was removed and then 50 *μ*L dimethyl sulfoxide (DMSO) was added. After shaking for 10 min at 37°C, the absorbance of each well was measured at a wavelength of 595 nm with a Bio-Tek microplate reader (Winooski, VT, USA). Experiments were designed in a triplicate format and cell proliferation rates were expressed as percentage proliferation compared to controls.

### 2.8. Wound Closure Migration Assay

Cells (5 × 10^5^/well) were seeded in a 24-well plate and cultured to reach confluence and then scraped with a sterile micropipette tip to create a denuded zone (gap) with a constant width (*T*_0_). After removing cell debris with repeated PBS rinses, fresh serum-free DMEM medium with or without P4 (30 ng/mL) and/or other testing reagents were supplemented. Anti-mPR*α* antibody (1 : 200) and/or anti-mPR*α* blocking peptide (1 : 100) were added two hours before P4 treatment. PP1 (10 *μ*M), AG 1478 (1 *μ*M), wortmannin (0.1 *μ*M), rapamycin (10 nM), and BpV (phen) (1 *μ*M) were added one hour before P4 treatment. The cells migrated at various speeds toward the middle axis from both edges of the scraped gaps, depending upon the treatment of aforementioned testing reagents, when they were incubated continually for 16 hours. After incubation, the width of the gap (*T*_16 hrs_) was measured by Image J. The rate of wound closure (WC) was calculated by the following equation: WC = 1 − (*T*_16 hrs_/*T*_0_)∗100% [53]; as referring control cells, migration inhibiting rate of treated cells (MIR) = 1 − (WC_treatment_/WC_control_)∗100%.

### 2.9. Invasion Assay

Cell invasion was assayed using the BD BioCoat Matrigel Invasion Chamber (BD Biosciences, MD, USA) [54]. Cells (4 × 10^4^ cells/well) were seeded in the upper chamber of a 24-well BD transwell coated with Matrigel and cultured with DMEM medium containing 1% FBS. After treatment with P4 at 30 ng/mL for 24 hrs with or without PP1 treatment at 10 *μ*M for one hour, the complete medium was applied to the lower chamber as chemoattractant. Cells were washed by PBS and then incubated for additional 16 hrs and the cells in the upper surface of the chamber membrane were then carefully removed with a cotton swab. Cells that invaded into the lower surface of the membrane were fixed with 10% buffered formalin and stained with hematoxylin solution. The number of invading cells (IC) from twenty random microscopic fields (×200 magnification) was counted. Invasion inhibition rate (IIR) was calculated as follows: IIR = 1 − (IC_treatment_/IC_control_)∗100%.

### 2.10. Statistical Analysis

The data was expressed as mean ± standard error (SE) and statistical differences between mean values were determined by Student's paired two-tailed *t*-test, followed by Fisher's protected least significance difference (PLSD). *P* < 0.05 was considered significant.

## 3. Results

### 3.1. Upregulation of mPR*α* Expression in the Brain Seeking MB231Br Cells

The brain seeking MB231Br cell line is increasingly used as a work horse model in brain metastatic studies, even though the molecular basis for its brain metastatic tropism is largely unknown [47, 48]. It was suggested that these cancer cells acquire the capacity to colonize brain* in vivo* following alternations in gene expression [47, 48]. In this study, we found that the expression of mPR*α* was upregulated from underdetectable to moderately positive at both the transcriptional and translational levels. As shown in Figure 1(a), the designated PCR band for mPR*α* in MB231Br cells was clearly seen at a moderate level (line 1), while there was no band for the parent MB231 cells (line 2) and there were very strong bands for the mPR*α* cDNA transfected MB231 cells and MB468 cells (lines 3 and 4). Using cell lysates isolated from those cells, an identical pattern of mPR*α* protein expression was documented by Western blot assays (Figure 1(b)). To determine if mPR*α* protein in MB231Br cells is translocated to the membrane compartment, we performed* in vitro* binding tests using a cell impermeable P4 conjugate (P4-BSA-FITC). After a short incubation (30 min), we observed clear fluorescent signals in the membrane of MB231Br cells (white arrows, Figure 1(c)(A)). Similar fluorescent signals were also seen in the membrane of the mPR*α* transfected MB231 cells (Figure 1(c)(C)), but not in the parent MB231 cells (Figure 1(c)(B)). To further demonstrate the binding specificity, we coincubated MB231Br cells with P4-BSA-FITC conjugate and excessive unconjugated free P4. As shown in Figure 1(c)(D), no fluorescent signals were shown in MB231Br cells. Binding studies with the fluorescent probe P4-BSA-FITC, which cannot enter cells because of the bulk moiety of BSA, confirms the presence of progestin-binding sites on the surface of cell membranes. This binding is specific because only free P4 was able to displace P4-BSA-FITC from breast cancer cells. This specificity was also confirmed by other studies that only unlabeled P4 human was able to substitute P4-BSA-FITC in pregnant myometrial cells* in vitro* whereas E2 and 11-deoxycortisone were ineffective [24, 25]. To study the function of mPR*α* receptor in MB231Br cells, we treated the cells with P4 at a series of concentrations (0, 30, and 60 ng/mL) for 48 hrs and demonstrated that the cell proliferation was inhibited in a dose dependent manner (Figure 2(a)). Cell morphological study showed that MB231Br cells without P4 incubation showed apparent mesenchymal phenotypes (Figures 2(b) and 2(c)), characterized by diverse sizes and spindle or elongated shapes, while, with P4 treatment, most of the cells showed epithelial-like phenotypes, featured by large and polygonal shapes or small oval shapes (Figures 2(d) and 2(e)).

### 3.2. Cell Migration of Human BPBC Cells in Response to Treatment of P4 and/or PP1

Further experiments were done to determine the effect of P4 treatment on cell migration. Using a wound closure assay, we found that the wound closure (WC) of MB231Br cells was slower (even though only marginally significant) when the cells were treated with P4 (30 ng/mL) for 16 hrs as compared to the cells without P4 treatment (40.6 ± 2.7% versus 50.0 ± 0.6%, MIR 18.9%, *P*_WC_ = 0.06, Figure 3). To explore the pathways that may be associated with P4's effect, the cells were coincubated with P4 and/or a number of pathway inhibitors. As shown in Figure 3, the WC rate for cells treated by Src1 inhibitor (PP1) alone was minimally inhibited (MB231Br cells 35.7 ± 8.9% versus 50.0 ± 0.6%, MIR 28.5%, *P*_WC_ = 0.11), which was comparable to cells treated with P4 alone (P4 versus PP1 *P* = 0.46). Coincubation of P4 and PP1 resulted in a significant lower WC rate, as compared to the control (9.7 ± 4.5% versus 50.0 ± 0.6%, MIR 80.6%, *P*_WC_ = 0.01) or to P4 or PP1 treatment alone (*P*_WC_ = 0.007 or 0.02). In addition, coincubation of P4 and PP1 also caused the lowest WC rates in MB468 cells (16.7 ± 1.5% versus 51.1 ± 1.5%, MIR 67.3%, *P*_WC_ = 0.001) and mPR*α* cDNA transfected MB231 cells (11.5 ± 0.6% versus 37.9 ± 2.9%, MIR 69.6%, *P*_WC_ value 0.009, Figure 3). In parental MB231 cells, neither P4 alone nor P4 in combination with PP1 treatment showed significant changes in wound closure rates as compared to that of control (P4, PP1, and P4 + PP1 versus control = 45.7 ± 0.6%, 44.8 ± 1.5%, and 43.3 ± 0.6% versus 45.6 ± 2.3%, all *P* values > 0.05, Figure 3). These results indicated that P4 + PP1 synergistically inhibit cell migration of mPR*α*+ human BPBC cells, namely, MB231Br, MB468, and mPR*α* cDNA transfected MB231 cells.

The mPR*α* expressing MB231Br cells were also treated with P4 and other pathway inhibitors, such as the EGFR inhibitor AG 1478 (51.7 ± 1.9%), PI3K inhibitor wortmannin (48.6 ± 0.5%), the mTOR inhibitor rapamycin (49.6 ± 1.2%), and the PTEN inhibitor (BpV (phen)) (47.8 ± 3.7%). There were no obvious WC differences observed as compared to controls (MIR were 2.2%, 3.8%, 1.7%, and 5.4%, *P* values were 0.80, 0.66, 0.84, and 0.63, respectively, Figure S1) (see Supplementary Material available online at http://dx.doi.org/10.1155/2014/426429).

### 3.3. MPR*α* and Its Role in Cell Migration of the Brain Seeking MB231Br Cells

In order to clarify the role of P4 → mPR*α* signaling in cell migration, we preincubated MB231Br cells with anti-mPR*α* antibody to block the binding of P4 to mPR*α* receptor one hour before P4 + PP1 cotreatment. The inhibitory effects of P4 + PP1 on cell migration were abrogated (WC 46.8 ± 3.3% versus 47.5 ± 3.7%, MIR1.5%, *P*_WC_ = 0.82), indicating that mPR*α* receptor plays a key role in P4 + PP1 induced cell migratory inhibition. When the cells were preincubated with anti-mPR*α* antibody and excess anti-mPR*α* blocking peptide, the inhibitory effects of P4 + PP1 on cell migration of MB231Br cells were restored (17.7 ± 2.3% versus 47.5 ± 3.7%, MIR 62.7%, *P*_WC_ = 0.001, Figure 4(a)).

### 3.4. Cell Invasion of the Brain Seeking MB231Br Cells in Response to P4 and/or PP1 Treatment

As cancer invasion* in vivo* is a three-dimensional process involving transendothelial migration and penetration through extracellular matrix, a 3D cell invasion model could further delineate the role of P4 and/or PP1 on metastatic potential of MB231Br cells [55]. To assess the role of P4 and PP1 on cell invasion of MB231Br cells, a cell invasion assay was performed. After P4 and/or PP1 treatment for 16 hrs, the number of cells that invaded into the lower chamber of Matrigel (IC) was decreased as compared to control (71 ± 2 versus 125 ± 1 cells, IIR 43.2%, *P* < 0.001), but treatment with either P4 or PP1 alone was ineffective (121 ± 4 and 116 ± 1 cells, IIR were 3.2% and 7.2%; *P*_IC_ values were 0.61 and 0.22). In parent MB231 cells, there were no obvious IC changes with or without P4 and/or PP1 treatment, as expected (Figure 4(b)).

### 3.5. Neither Nuclear PR Nor PGRMC1 Plays a Key Role in Mediating P4 + PP1's Inhibitory Effects on Cell Migration of MB231Br Cells

The expression of PR in basal phenotype breast cancer cells (i.e., MB468 cells) may be induced by P4 treatment, even though the extent of induction is very low [23]. To clarify if induction of endogenous PR expression has a role in the P4 induced cell migratory inhibition, we preincubated MB231Br cells with MIF, a PR antagonist, before P4 and/or PP1 treatment. It was found that wound closure rates were not affected after P4 and/or PP1 treatment (P4 versus MIF + P4, PP1 versus MIF + PP1, and P4 + PP1 versus MIF + P4 + PP1 were 38.9 ± 1.8% versus 35.3 ± 5.1%, 26.6 ± 4.2% versus 36.1 ± 5.6%, and 9.7 ± 4.5% versus 14.2 ± 4.9%; all *P*_WC_ values > 0.05, Figure 5(a)).

In addition to mPR*α*, PGRMC1 has been implicated in membrane-initiated progesterone signaling [56]. It is unclear whether mPR*α* functions alone or requires PGRMC1 as a comediator. In a Western blot assay, the protein expression of PGRMC1was observed noticeably in MB231Br cells but showed minimal changes with P4 and/or PP1 treatment (Figure 5(b)). We then preincubated MB231Br cells with PGRMC1 antibody to block or interfere with the function of PGRMC1 protein one hour before P4 and/or PP1 treatment. The wound closure rates, in the presence of anti-PGRMC1 antibody, demonstrated no change on cell migration pattern as compared to those induced by P4 alone or by P4 + PP1 (WC 15.2 ± 6.1% and 10.2 ± 1.4% versus 37.3 ± 3.4%, *P* values were 0.047 and 0.008, resp.). Treatment of anti-PGRMC1 antibody alone had no effect on cell migration (37.8 ± 4.3% versus 37.3 ± 3.4%, *P* = 0.93).

### 3.6. Molecular Pathways Involved in the P4 + PP1 Inhibited Cell Migration of MB231Br Cells

Based upon the results of cell migration assays, synergistic effect of P4 and PP1 on cell migration and invasion of MB231Br cells was suggested. Moreover, P4 has been reported to signal via Src family kinases for the formation of focal adhesion complex via focal adhesion kinase (FAK, a key component for tumor metastasis) phosphorylation at Tyr (397) [57]. To confirm the molecular mechanisms underlying P4 + PP1's action, we evaluated the phosphorylation of Src and FAK using Western blot assay. It was found that the level of phosphor-FAK in MB231Br cells was inhibited by P4 + PP1 treatment significantly (as compare to that of control, 43.6% versus 100%, *P* = 0.009), while the status of Src phosphorylation was not changed by P4 + PP1 cotreatment. P4 or PP1 treatment alone did not change the levels of phosphor-FAK in MB231Br cells (94.68%, 81.1% versus 100%, all *P* values > 0.05) (Figure 6(a)). We also investigated the effect of P4 and/or PP1 on expression of other selected cancer metastasis relevant proteins, such as MMP9, VEGF, and KCNMA1 [58]. The expression levels of MMP9 (79.3% versus 100%, *P* = 0.009), VEGF (33.2% versus 100%, *P* = 0.04), and KCNMA1 (77.6% versus 100%, *P* = 0.02) were reduced by P4 + PP1 cotreatment in MB231Br cells remarkably but again not by P4 or PP1 individual treatments as compared to controls (All *P* values > 0.05, Figure 6(b)).

## 4. Discussion

### 4.1. Upregulation of MPR*α* May Contribute to the Brain Metastatic Tropism of MB231Br Cells

The role of progesterone (P4) in breast cancer development has attracted substantial interest. It is believed that the physiological action of P4 is mediated through either nuclear PR or membrane-bound receptors. In this study, using RT-PCR and Western blotting assays, we first showed the expression of mPR*α* in the membrane of MB231Br cells, a functional site of this hormonal receptor. To study the function of mPR*α* in MB231Br cells, we demonstrated that P4 treatment inhibits cell proliferation (Figure 2(a)) and reverses cell morphology from mesenchymal phenotypes to epithelial-like phenotypes (Figures 2(b)–2(d)), while in mPR*α* negative MB231 cells P4 treatment had no effect. These results were consistent with our previous results on MB468 cells [23]. Khan et al. performed a genowide expression profiling on two human BPBC cell lines—parental MB231 and brain seeking MB231Br cells [59]. They found elevated levels of genes that promote cell motility and invasion, while genes that prevent cancer metastasis were downregulated in MB231Br cells (compared to parental MB231 cells) [60–62]. Bos et al. compared the gene expression profiles of the brain seeking cells from MDA-MB-231 and CN34 cells from the tumor of an ER-patient [50]. They found 243 genes differentially expressed between the brain metastasis and parental cell lines. Of those, the expression of 17 genes was correlated with brain relapse in patient samples without association with bone, liver, or lymph node metastasis [63]. It was assumed that these altered gene expression profiles acquainted from a series of* in vivo/ex vivo* selections may facilitate the successful colonization in brain.

### 4.2. MPR*α* May Serve as a Key Mediator for P4's Action on Cell Migratory and Invasion Inhibition in MB231Br Cells

Progesterone is known to play a profound role in breast cancer cell migration. In this study, we showed that P4 treatment alone can slightly inhibit, rather than enhance, the cell migration of MB231Br cells; more interestingly, treatment of P4 plus PP1 can significantly inhibit cell migration of MB231Br cells. Since PP1 treatment alone inhibited cell migration only at a moderate level, which was comparable to P4, we assumed that combinational treatment with both can synergize the molecular signal magnitude and vigorously inhibit cell migration* in vitro*. Similarly, in cell invasion assay, synergistic results were also obtained from the cells which were treated by P4 + PP1 (IIR 43.2%) but not by P4 or PP1 alone (IIR = 3.2% and 7.2%), while Fu et al. found that cell migration and invasion were both enhanced by all the P4 and its derivatives tested in T47-D cells (ER+/PR+) [64, 65]. Different results may be due to various cell lines with different PR and ER expression.

Since parent MB231 cells do not contain full-length or C-terminus PRs [66], we assumed that the acquired expression of mPR*α* may serve as a key mediator for P4's action in MB231Br cells. This assumption was supported by the following findings. (1) Block the binding of P4 to mPR*α* receptor by preincubating MB231Br cells with anti-mPR*α* antibody, which abrogated the inhibitory effects of P4 + PP1 on cell migration. Preincubating the cells with anti-mPR*α* antibody and excess anti-mPR*α* blocking peptide, the inhibitory effects of P4 + PP1 on cell migration were unaffected. These results indicated that the role of mPR*α* in cell migration and regulation is essential. (2) P4 treatment may upregulate PR expression in human BPBC cells (e.g., MB231 cells) [23, 67], which could mediate the effect of P4. To exclude the potential role of PR in this study, we preincubated the cells with MIF, a P4 antagonist, and found that it did not affect P4's and/or PP1's effects on MB231Br cell migration. (3) PGRMC1 is required for some aspects of P4 signaling in estrogen receptor-negative breast tumors through an unidentified mechanism [68, 69]. Thomas et al. demonstrated that overexpression of human PGRMC1 in nuclear PR negative breast cancer cell lines causes increased expression of mPR*α* on cell membranes and increased specific P4 binding [70]. To exclude the potential role of PGRMC1 in this study, we demonstrated that P4 and/or PP1 treatment had no effect on PGRMC1 expression in MB231Br cells, as compared to that in vehicle treated control cells. In addition, coincubating the MB231Br cells with anti-PGRMC1 antibody and P4 and/or PP1 did not affect the cell migration patterns. These results suggested that PGRMC1 and its signaling pathways may not be involved in the roles of P4 and PP1 on cell migration.

### 4.3. Molecular Pathways Involved in P4 + PP1/mPR*α* Signaling

Progesterone exerts rapid nongenomic actions which are triggered by P4 binding to mPR*α* [34–36] and subsequently induces a series of alterations in secondary messenger pathways through activation of pertussis toxin-sensitive inhibitory G-proteins, to activate MAPK/Erk 1/2 pathway [32, 33, 37, 38]. We recently reported that the signaling cascade of P4 induced mesenchymal repression of human BPBC cells through caveolae bound signaling molecules, namely, Cav-1, EGFR, and PI3K. We also observed that the Src family kinase inhibitor (PP1) blocked the P4's action on proteins that control cell epithelial differentiation but not on the proteins that control cell mesenchymal differentiation. Src has been reported to be a starting point for many biochemical cascades and exerts a profound effect on focal adhesion systems and cytoskeleton reorganization and thereby influences cancer cell migration and invasion as well as other tumor progression-related events [71]. In this report, we showed that P4 + PP1 (a Src family inhibitor [72, 73]) synergistically inhibited the cell migration of the mPR*α* expressing MB231Br cells significantly. Focal adhesion kinase (FAK) is a downstream component of Src signaling pathway controlling cell motility [74]. Through multifaceted molecular connections, FAK controls cell movement by regulating the cytoskeleton structures, cell adhesion sites, and membrane protrusions [74, 75]. In presence of PR, P4 could induce the phosphorylation and activation of FAK [76]. For example, MB231 breast cancer cells transfected with PR were exposed to P4 and displayed an increased expression of phosphorylated FAK and formation of FA complexes, which led to an enhanced cell migration and invasion [76]. In human BPBC cell models, which are depleted of nuclear PR but mPR*α* positive, P4 and PP1 cotreatment induced significant FAK dephosphorylation (rather than phosphorylation), while P4 or PP1 individual treatment did not affect the status of FAK. This may explain the diverse roles of P4 in different human BPBC and non-BPBC cancer cells. Also, the roles of other pathway inhibitors on cell migration of MB231Br cells were also tested. Cotreatment of these cells with P4 and EGFR inhibitor (AG 1478) or PI3K inhibitor (wortmannin) or mTOR inhibitor (rapamycin) and/or PTEN inhibitor (BpV (phen)) had no obvious WC differences observed as compared to controls (Figure S1).

To determine the downstream effector protein molecules of Src/FAK pathway, we studied metastatic relevant protein expression profiles. Matrix metalloproteinases (MMPs) and VEGF have been implicated in several aspects of tumor progression, such as invasion through basement membrane and interstitial matrices, angiogenesis, and tumor cell growth. In the present study, we found that MB231Br cells express MMP-9 and VEGF at comparable levels as that of MB231 cells. In response to P4 or PP1 treatment alone, the expression of MMP9 and VEGF in MB231Br cells exhibited minimal changes; however, combination treatment with both induced significant reduction in MMP9 and VEGF expression, a similar pattern as that of FAK dephosphorylation, supporting these prometastatic proteins as the downstream effectors of Src/FAK pathway. KCNMA1 (large conductive calcium-activated potassium channel, subfamily M, alpha member 1) is a pore forming *α*-subunit of the large-conductance calcium- and voltage-activated potassium channel (BK_Ca_) [77]. KCNMA1 expression was reported in metastatic breast cancer cells and increased BKCa channel activity might associate with greater invasiveness and transendothelial migration [58]. It was assumed that the relative abundance of BKCa channel expression in brain metastatic breast cancer may provide a unique opportunity to identify breast tumors that are at high risk for brain metastasis [58]. In this study, we found that KCNMA1 expression was also inhibited in MB231Br cells in a similar pattern as compared with that of FAK dephosphorylation and MMP9 expression in response to P4 and/or PP1 treatment. We assumed that MMP-9 and KCNMA1 serve as terminal effects of the Src/FAK signal pathway.

## 5. Conclusions

In summary, using brain seeking MB231Br cells and other human BPBC cell lines as models, we identified an mPR*α* mediated pathway that involves Src/FAK and a chain of downstream cell signaling components. This molecular pathway could be inhibited by incubating MB231Br cells with P4 and PP1 concurrently. It was assumed that PP1 enhances the P4's effect on FAK dephosphorylation, MMP9, VEGF, and KCNMA1 downregulation and eventually inhibits cell migration synergistically. Our study has provided a mechanistic view on the effects of P4 as a promising physiological anticancer agent, through mPR*α* → Src/FAK relevant signal transduction pathways in human BPBC cells.

## Supplementary Material

Fig. S1. Effect of P4+PP1 on cell migration of MB231Br cells in presence of various pathway inhibitors.

## Figures and Tables

**Figure 1:** MPR*α* mRNA (a) and protein (b) expressions and receptor distribution (c) in various human BPBC cells. As shown in (a) and (b), the samples of mPR*α* mRNA and protein are indicated as “1–4,” representing MB231Br, MB231, mPR*α* cDNA transfected MB231 (231 w/mPR*α*), and MB468 breast cancer cells, respectively. The expressions of 18S and *α*-tubulin are used as references. (c)(A)–(c)(C) show the results of incubating the cells with P4-BSA-FITC conjugates (white arrows indicate the specific binding sites), MB231Br cells, MB231 cells, and MB231 cells w/mPR*α*, respectively; (c)(D) shows the result of incubating MB231Br cells with P4-BSA-FITC conjugates and excessive free P4. Images were taken under confocal microscope using ×60 oil objective lens.

**Figure 2:** Effect of P4 on cell morphology and proliferation of MB231Br. (a) shows the results of cell proliferation assay of MB231Br and MB231 cells (^∗^0.05 > *P* > 0.01). (b) and (c) show the cell morphology of MB231Br without P4 treatment; (d) and (e) show the cells treated by P4 (30 ng/mL and 60 ng/mL). Images were taken under confocal microscope (DIC) using ×40 oil objective lens.

**Figure 3:** Effect of P4 + PP1 on cell migration of human BPBC cells. The left panel shows the wound closure assays of MB231Br, MB231, MB468, and mPR*α* transfected MB231 cells (231 w/mPR*α*), with or without P4 and/or PP1 treatments. Images were taken under confocal microscope using ×10 objective lens. The right panel shows the summarized data from four independent assays (^∗^0.05 > *P* > 0.01 and ^∗∗^ *P* < 0.01).

**Figure 4:** (a) Effect of P4 + PP1 on cell migration of MB231Br in presence of anti-mPR*α* antibody and mPR*α* blocking peptide. (Ab/ppt: anti-mPR*α* antibody and mPR*α* blocking peptide.) The up panels of (a) show the wound closure assays of MB231Br and MB231 cells with or without treatments as indicated. Images were taken using confocal microscope (×10 objective lens). The low panel of (a) shows the summarized data from two independent assays (^∗∗^ *P* < 0.01). (b) Effect of P4 + PP1 on cell invasion of MB231Br. The left panel of (b) shows the cell invasion assays of MB231Br and MB231 cells with or without P4 and/or PP1 treatments as indicated. The right panel of (b) shows the summarized data from two independent experiments (^∗∗^ *P* < 0.01).

**Figure 5:** (a) Effect of P4 + PP1 on cell migration of MB231Br in presence of MIF. The up panels of (a) show the wound closure assays of MB231Br and MB231 cells with or without P4 and/or PP1 treatments as indicated. All of the cells were preincubated with MIF. Images were taken under confocal microscope using ×10 objective lens. The lower panel of (a) shows the summarized data from two independent assays (^∗^0.05 > *P* > 0.01). (b) Effect of P4 + PP1 on cell migration of MB231Br in presence of anti-PGRMC1 antibody. Growth-arrested MB231Br and MB231 cells were treated with or without P4 and/or PP1 treatment as indicated. Western blot assays for evaluating PGRMC1 expression were performed. The up panel of (b) shows the representative image from three Western blot assays. The middle panel of (b) shows the wound closure assays of MB231Br cells with or without P4 and/or PP1 treatments as indicated. Images were taken under confocal microscope using ×10 objective lens. The graph in the bottom of (b) shows the summarized data from four independent assays (^∗^0.05 > *P* > 0.01, ^∗∗^ *P* < 0.01).

**Figure 6:** Effect of P4 + PP1 on FAK phosphorylation and expression of MMP-9 and KCNMA1 in MB231Br cells. Growth-arrested MB231Br and MB231 cells were treated with or without P4 and/or PP1 treatment as indicated. Western blot assays for evaluating the status of Src and FAK phosphorylation and expression of MMP-9, VEGF, and KCNMA1 were performed with proper antibodies. The up panel shows the representative image from three Western blot assays. The graph in the bottom shows the summarized data from three independent assays (^∗^0.05 > *P* > 0.01).

## Abbreviations

BPBC: Basal phenotype breast cancers
P4: Progesterone
MB468: MDA-MB468 cells
EMT: Epithelial-mesenchymal transition
mPR*α*: Membrane progesterone receptor *α*
MB231: MDA-MB231 cells
PRs: Progesterone receptors
ATCC: American Type Culture Collection
IHC: Immunohistochemistry
TNBC: Triple negative cancers.
